The article "Children's Computation of Complex Linguistic Forms: A Study of Frequency and Imageability Effects" was published in 2013. Journal: PLoS One.

# Children's Computation of Complex Linguistic Forms: A Study of Frequency and Imageability Effects

**DOI:** 10.1371/journal.pone.0074683

**Published:** 2013-09-09

**Authors:** Cristina D. Dye, Matthew Walenski, Elizabeth L. Prado, Stewart Mostofsky, Michael T. Ullman

**Affiliations:** 1 Centre for Research in Linguistics and Language Sciences, Newcastle University, Newcastle Upon Tyne, Tyne and Wear, United Kingdom; 2 Brain and Language Lab, Department of Neuroscience, Georgetown University, Washington, DC, United States of America; 3 School of Speech, Language, and Hearing Sciences, San Diego State University, San Diego, California, United States of America; 4 Center for Research in Language, University of California San Diego, San Diego, California, United States of America; 5 Department of Nutrition, University of California Davis, Davis, California, United States of America; 6 Kennedy Krieger Institute, Johns Hopkins University, Baltimore, Maryland, United States of America; Stony Brook University, United States of America

## Abstract

This study investigates the storage vs. composition of inflected forms in typically-developing children. Children aged 8–12 were tested on the production of regular and irregular past-tense forms. Storage (vs. composition) was examined by probing for past-tense frequency effects and imageability effects – both of which are diagnostic tests for storage – while controlling for a number of confounding factors. We also examined sex as a factor. Irregular inflected forms, which must depend on stored representations, always showed evidence of storage (frequency and/or imageability effects), not only across all children, but also separately in both sexes. In contrast, for regular forms, which could be either stored or composed, only girls showed evidence of storage. This pattern is similar to that found in previously-acquired adult data from the same task, with the notable exception that development affects which factors influence the storage of regulars in females: imageability plays a larger role in girls, and frequency in women. Overall, the results suggest that irregular inflected forms are always stored (in children and adults, and in both sexes), whereas regulars can be either composed or stored, with their storage a function of various item- and subject-level factors.

## Introduction

How is language computed in the mind? Although we now know that language computation requires both storage and composition, it remains unclear which aspects of language are stored and which are (de)composed, and under what circumstances. Moreover, this is even less well understood in children than adults. In adults, a considerable amount of research has investigated this issue by probing for storage effects in the on-line computation of existing inflected forms, in particular in the contrast between regular and irregular inflected variants (e.g., *walked* vs. *dug*), which can be equated for phonological, semantic, and other factors. Here, we examine this issue in children.

### Storage/composition theoretical models

A variety of theoretical proposals regarding the computation of existing inflected forms have been put forth. These can be grouped in two broad classes: single-mechanism models and dual-system models.

Single-mechanism models propose that all inflected forms are computed with the same basic mechanisms. For example, according to connectionist models, all previously-encountered inflected words are represented in a distributed associative memory [1]–[6]. Such models suggest that forms that exhibit a common and consistent inflectional pattern (regular forms, as well as some irregulars, such as *sing-sang, ring-rang*) rely primarily on phonological representations in this distributed memory. Rule-only models constitute another type of single-mechanism model. Here, too, all inflected forms (i.e., both regular and irregular) are handled by the same or similar mechanisms, which in this case, involve rule-based processes [7]–[10].

Dual-system models, on the other hand, hold that while some inflected forms are stored, the computation of others depends on (de)composition by rule-governed processes in a separate computational and neurocognitive system. Irregularly inflected forms (e.g., *dug*), which cannot be fully specified by a default rule, are claimed to depend on memorized representations. Regulars hold a different status. Some dual-system models hold that regulars are always composed (e.g., *walk +ed*) by a default rule [11]–[13]. Others, however, suggest that even if regulars can be assembled by rule-governed processes, they can also be stored, and indeed often are, with the likelihood of storage depending on various item-level (e.g., frequency) and subject-level (e.g., sex) factors [14]–[20]. For example, women, who appear to have superior verbal memories as compared to men [21]–[25], may also be more likely than men to store regularly inflected forms [14], [20], [25].

These models, as well as similar ones, have been proposed not only for adults, but also for children. Models claiming the dependence of all inflected forms on (an associative) memory suggest that children, like adults, rely on word storage or pattern association for both regulars and irregulars. For example, Bybee [26], [27] suggests that the child memorizes specific verb items (whether regular or irregular forms), and forms networks of associations among them, which eventually reveal common subparts (e.g., *play* in *plays* and *playing*) and allow for generalization of common inflection patterns by analogy. Connectionist models also emphasize the dependence of all the child's forms (regardless of regularity type) on memory [5], [28]–[30]. Rule-only models suggest that children would gradually induce multiple rules from the lexicon through ‘minimal generalization’ [7].

Dual-system models have taken a different approach to the development of the representation and computation of inflected forms. Children are thought to initially memorize both regular and irregular inflected forms (e.g., *talked, dug*), though by an early age, e.g. by around age 3 for English past-tense, they acquire the appropriate rule(s) – as evidenced, for example, by their fairly consistent *–ed* affixation not only of regulars (e.g., *talk-talked*), but also of nonce verbs (e.g., *rick-ricked*), and even irregular verbs, resulting in over-regularizations such as *goed* or *eated* [31]–[33]. Thus, at least after a very early age, children are thought to compute inflected forms in a qualitatively similar way to adults – that is, depending on both storage and composition, even though the extent to which each of these may be relied on may differ between children and adults. For example, the fact that adults hardly ever over-regularize [31], [34], is explained on a dual-system view by the tendency for children to have been exposed to fewer irregularly-inflected forms than adults; children thus have weaker memory traces for irregulars than adults, making it more likely for a child to fail at retrieving an irregular form from memory and thus less likely to resort to rule-based composition and over-regularizations [31].

### Frequency effects and imageability effects as diagnostic tests of storage

In the current study we use two related techniques to investigate the storage vs. composition of existing (real) regular and irregular English past-tense forms in children. These two techniques – probing for frequency effects and for imageability effects – can help distinguish between storage and composition, and can therefore be used to test predictions made by various models with respect to this distinction.

The method of probing for “frequency effects” is based on the fact that lexical forms that are more frequently encountered are also more rapidly or more successfully accessed in memory than forms encountered with lower frequency, findings which hold for both adults and children [35]–[39]. If inflected forms are stored, they should exhibit such frequency effects. That is, such forms should show correlations between their inflected-form frequencies and measures of their accessibility (e.g., response times). In contrast, inflected forms that are composed rather than stored should not exhibit such correlations, once access to their stems is controlled for. The presence of frequency effects therefore can and has been used as a diagnostic test of the storage of inflected forms.

A second and more recent method for investigating the storage of lexical forms involves probing for “imageability effects” [20]. The logic of imageability effects is based on the well-documented finding that, in adults as well as children, lexical items for which a visual mental image is more easily formed are also more easily memorized and accessed than forms that are harder to visualize [40]–[49]. Therefore, stored forms, including stored inflected forms, may be expected to exhibit imageability effects: that is, correlations between their imageability and measures of their accessibility. For example, if irregular past tense forms are stored, those of verbs with higher imageability (e.g., *dug*) should be better memorized and thus accessed faster than those of verbs with lower imageability (e.g., *thought*), regardless of the fact that their (stored) stems should also show this effect. Such imageability effects should hold even when stem access is controlled for (e.g., by presenting the stems to subjects in a production paradigm). In contrast, inflected forms that are composed would *not* be expected to show imageability effects (e.g., *walked* vs. *balked*), once access to their stems is controlled for. Note that if lexical access to stems rather than past-tense forms was in fact driving imageability effects in past-tense production, we would expect to see imageability effects on *all* past-tense forms, including forms that are posited to be composed (e.g., regulars in males); as we will see however, this is not the case, either in the present study or for previous findings [20]. Thus imageability effects on inflected forms seem to be due to the retrieval of those forms rather than their stems (even though the imageability of stems and past-tense forms are likely to be the same or very similar). In sum, inflected forms that are stored should exhibit imageability effects in addition to or instead of frequency effects (depending on which of these factors has the greatest influence), allowing imageability effects to be used as another diagnostic of storage.

It should be noted that whereas proponents of different theoretical views largely agree that the presence of frequency effects is indicative of storage [50], there is less consensus concerning the interpretation of an absence of frequency effects (imageability effects are a new diagnostic, and have not been discussed in this respect, but one may expect a similar argument to apply). Single mechanism proponents have argued that a lack of frequency effects on certain inflected forms need not necessarily indicate that these forms are not stored. For example, given that all regulars have a similar stem-past phonological transformation, this generalized phonological pattern is thought to be learned in associative memory, leaving little or no influence for the frequencies of individual past-tense forms. In this case the contribution of neighboring (i.e., phonologically similar) regulars to a given verb's memory traces may overwhelm the contribution of each verb's individual past tense frequency, resulting in weakened past tense frequency effects for regulars [28], [29], [51].

In contrast, proponents of dual-system models claim that inflected forms that depend on composition rather than storage are not expected to exhibit frequency effects, once confounding factors, including phonological similarity to other verbs, are controlled [52], [53]. On this view, irregularly inflected forms should always show signs of storage (e.g., from frequency and/or imageability effects), whereas regulars should show storage in *some* circumstances but *not* others (e.g., for females but not for males). Importantly, this particular pattern of predictions has not been made by single-mechanism models, allowing the two types of models to be potentially distinguished.

### Previous evidence from adults

Most studies of frequency effects on existing inflectional forms have focused on adults. A number of studies have reported frequency effects for irregular but not regular inflected forms. This pattern of results has been observed for English past-tense forms [6], [20], [52], [54], [55], German noun plurals [56], [57], German past participles [58], and French verb forms [59]. Consistent with this pattern, a lack of frequency effects has also been reported for regular inflected forms in Dutch [60]. However, other studies have reported frequency effects for regular inflected forms, for example in English noun plurals [61], English past tense forms [6], [62], Finnish noun plurals [63], and Dutch verb forms [53].

These discrepant findings for regular inflected forms may be explained by a range of item and subject-level factors that may influence the storage of regulars. Results from several studies support this view, and have revealed that only certain types of regulars show frequency effects, or certain subject groups show frequency effects on regulars. For example, frequency effects have been observed for higher-frequency (but not lower-frequency) regular forms in a number of studies, including in English regular past-tense forms [3], [15], [20], Dutch noun plurals [16], Swedish definite nouns [17], and Finnish (genitive, locative, and partitive) nouns [18], [19]. Of particular interest in the current study, frequency effects on regulars have been observed in women but not men for English past tense forms [20], and were found to be stronger in women than men for Danish noun, verb, and adjective forms [64].

To our knowledge, imageability effects on the processing of inflectional morphology have been examined thus far in only one study, Prado and Ullman (2009) [20], which found imageability effects for irregular but not regular past-tense forms among men. In contrast, imageability effects were not observed for women on either regulars or irregulars [20]. See Discussion below.

### Previous evidence from children

In children, who represent the focus of the current investigation, only a handful of empirical studies of frequency effects on existing (i.e., not nonce) inflected forms have been carried out, and no studies have examined imageability effects. The findings with regards to frequency effects on regular forms have been somewhat mixed. One study of frequency effects on the processing of inflected forms in British English [65] examined accuracy rates in the production of regular and irregular past-tense forms in 36 typically-developing children ages 5;5 to 8;9 (as well as children with Specific Language Impairment, not discussed here). Frequency effects were observed for irregulars but not regulars. Similar results were obtained in a study on German past participles, in which reaction times were obtained from 40 children between 5 and 12 years old, all of whom listened to verb stems and were asked to produce corresponding past participle forms [58]. Again, frequency effects were found for irregulars but not for regulars. In contrast, two studies have reported frequency effects on either both [66] or neither [67] regulars and irregulars. A study of 15 Quebec French-speaking children aged 2;11 to 4;6 reported frequency effects on accuracy across *both* regular and irregular past tense (passé composé) forms [66]. In contrast, a study of 18 British English-speaking children, mean age 11, found *no* frequency effects on response times across regular and irregular past-tense forms [62]. Finally, a recent study of 307 British English-speaking 4–8 year old children investigating frequency effects in noun plurals and past tenses found inconsistent frequency effects for both regulars and irregulars across age groups though the dependent variable (percentage of responses with inflected forms) collapsed together correctly inflected and over-regularized responses, making it difficult to assess the results with respect to correctly inflected forms [67]. Note that studies of children's production of nonce or overregularized forms (or other errors) [31], [68]–[72] are beyond the scope of the present study, which focuses on the computation of *correct existing* forms.

Although these previous studies of frequency effects constitute important initial steps in the investigation of the storage/composition distinction of inflected forms in children, they do not take into account a number of issues, some or all of which may have contributed to inconsistencies across the results. First, no prior study on children has examined imageability effects. Given that imageability effects have been shown to be a useful diagnostic of storage in adults [20], investigating imageability effects in children may shed light on the storage versus composition of inflected forms at younger ages as well. Second, previous studies of children have not explored the role of subject-level factors such as sex. Given that sex has been found to influence frequency as well as imageability effects in adults [20], [64], this factor should also be examined in children. Analyses stratified by sex might help explain potential frequency or imageability effects on regulars, and may explain at least some of the inconsistencies across previous results. Methodologically, frequency has previously been treated as a dichotomous variable in most studies, divided into ‘high’ and ‘low’ frequency groups. This dichotomization may have led to degraded measurement and loss of power [73], [74]. Additionally, the data have generally been averaged over subjects and responses, a technique that has similar consequences [73], [74]. Statistical techniques such as those used in the current study avoid this loss of power and therefore could lead to the detection of frequency effects where they might have remained undetected in previous studies.

### The Current Study

Here we investigate children's storage vs. composition of existing English past-tense forms by examining both frequency and imageability effects, as well as the possibility of sex differences with regard to these effects. Methodologically, we use approaches that avoid the loss of power entailed by using averaged data and dichotomizing continuous variables, and we control (experimentally and/or statistically) for a large number of potentially confounding factors. Finally, we provide direct comparisons with adult data in order to probe for developmental changes between boys and girls and adult men and women.

## Methods

### Subjects

We tested forty-five healthy right-handed monolingual North American English-speaking children (8–12 years old, mean age  = 9.67, *SD* = 1.35; 22 girls) from the greater Washington DC area. The age range for the children was selected a priori based on the following considerations: a) we wanted to examine children who are past what is traditionally considered the age of overregularization [31], and b) the age range was similar to the age ranges in previous work investigating frequency effects on the production of past-tense forms in children [58], [62]. The children had a mean of 4.6 years of education (*SD* = 1.4). Handedness was assessed based on the Edinburgh questionnaire [75]. All children had normal or corrected-to-normal hearing and vision, and none had any known history of developmental, psychiatric or neurological disorders. Ten children produced correct answers for fewer than half of the items of either verb type (regular and irregular). Since only response times to correct answers were analyzed (see below), these children were excluded to avoid insufficient data points from any child (note that including these ten children in the analyses yielded an almost identical pattern of findings). The remaining 35 children (8–12 years old; mean age  = 9.91, *SD* = 1.38; 16 girls) had a mean of 4.89 years of education (*SD* = 1.47). Children were also tested on the Reading section of the Wechsler Individual Achievement Test Second Edition (WIAT-II) [76] and scored within the normal range (two of the 35 children analyzed did not complete this test). Reading scores for girls (*M* = 118.2, *SD* = 8.81) did not differ statistically from those for boys (M = 112.1, *SD* = 11.36, t(31)  = 1.69, *p* = 0.100).

In addition, we directly compared the data from the children to data from 71 adults (18–50 years, mean age  = 24.97, *SD* = 7.83; mean 15.34 years of education, *SD* = 1.79; 35 women), whose frequency and imageability effects were previously reported in Prado and Ullman (2009) [20]. All adults met the same language, handedness, and neuropsychological criteria as the children.

### Ethics statement

This study was approved by the Georgetown University Institutional Review Board. Children's parents provided written consent and children provided oral assent, which was documented by the experimenter on the consent form at the beginning of the test session.

### The Past Tense Production Task

Subjects were tested on a past tense production task that has been described in detail in previous literature [20], [77]. In summary, we examined subjects' performance on the production of 29 irregular verbs (e.g., *hold-held*), and 29 regulars (e.g., *fail-failed*: these did not include inconsistent regulars, whose stems are phonologically similar to the stems of irregulars, e.g., *squeeze-squeezed*, whose stem is similar to *freeze-froze*). The test items did not include any no-change verbs (e.g., *hit-hit*) or any verbs for which both a regular and an irregular past-tense are acceptable (e.g., *dive-dived*/*dove*). The 29 regulars and 29 irregulars were matched group-wise on the following measures (further described below): stem (uninflected form) frequency, past-tense frequency, and imageability (paired *t*-tests, *p*s>.40).

To quantify past-tense *frequency* (and stem frequency), two counts were used in combination: (1) a frequency count extracted by a stochastic part-of-speech analyzer from a 44 million word corpus of unedited Associated Press news wires [52], [78] (AP); and (2) the Francis and Kucera [79] count (FK), derived from a 1 million word corpus composed of a variety of sources. All analyses were carried out on the natural logarithm of the sum of the two frequency counts, first augmented by 1 to avoid the undefined ln(0).

These frequency counts were chosen for several reasons. First, frequency counts from large corpora are highly desirable because they provide much greater signal than those from small corpora. Since it was crucial to have large corpora, it was not possible to use corpora specifically involving children in the relevant age range, which are typically much smaller in size. Second, this decision is also in line with previous studies, which have likewise used adult frequency counts in work with children in the same age range as our subjects [58], [62], [65]. Third, it has been shown that verb familiarity ratings obtained from children in this age range correlate with adult frequency counts [65]; additionally, frequency counts based on child-addressed speech as well as child speech correlate with adult frequency counts [58]. It might be argued that the potential inappropriateness of adult frequency counts for children could lead to a high likelihood of false negatives for children's frequency effects. However, in the present study children did *not* in fact show weaker frequency effects than adults on irregulars (which must be stored), suggesting that the adult frequency counts employed here are sufficient to detect frequency effects in the children examined in this study.

Only verbs that were likely to be known by 8-year-olds were included, as determined by the unanimous judgments of five adult native speakers of North-American English, based on the procedure described in [38]. Additionally, note that the children in our study responded accurately enough for us to detect frequency effects on irregulars, and were even more accurate on regulars (see Results).

The *imageability* ratings, which were taken from Prado and Ullman (2009) [20], ranged from 1 (low imageability) to 5 (high imageability). As in previous studies of imageability in children [38], [80], the present study used imageability ratings obtained from adults. Although it might be argued that the use of adult imageability ratings as a predictor for both age groups might lead to a higher likelihood of false negatives in children than adults (i.e., weaker imageability effects in children), in fact the only reliable difference between children and adults found for imageability effects (on regulars) was *more* reliable in children (girls) than adults (women), arguing against such a confound (see Results).

The imageability ratings were based on the uninflected form of the verb (e.g., *dig, walk*), which was used as a proxy for the imageability of the past tense since, as a semantic property, imageability is not expected to differ between the uninflected form and the past tense form. The details of the methodology used for obtaining these imageability ratings are described in Prado and Ullman (2009) [20]. In brief, 28 subjects completed a paper and pencil task in which they were asked to rate a set of words, including the verbs used in the present investigation, in terms of their imageability (on a scale from 1 to 5). Half of the subjects who contributed the ratings were men and half women. Mean imageability ratings were computed for each item over all subjects. The imageability ratings across all regulars and irregulars did not differ between the males and females; additionally the regulars and irregulars did not differ in their imageability ratings. The obtained imageability ratings correlated with previously published imageability ratings.

#### Procedure

Each verb stem was presented alone and in the context of a sentence, with a second sentence containing a blank to elicit the past-tense form (e.g., *fail. Every day I fail an exam. Just like every day, yesterday I ____ an exam*), all displayed simultaneously on the computer screen [20]. The sentences were identical apart from the verb and the post-verbal material (which was composed of two words, neither of which was inflected or of low frequency). Items were pseudo-randomized, and item order was controlled for statistically (see below). Subjects were instructed to produce the missing form as quickly and accurately as possible. Response time (RT) data were recorded via a microphone connected to a computerized timer, and were measured from the time the sentence appeared on the screen to the time the subject initiated their response.

#### Analysis

Frequency and imageability effects were examined on RT data. During testing, the experimenter noted items where the RTs were not triggered by the subject's response; these response times were not analyzed. RT analyses were performed only on correct first-responses (94.29% of all first responses to the 58 regular and irregular verbs). Very fast responses, that is RTs faster than 500 ms, were discarded as being likely due to computer error (3.64% of non timer-error correct responses). Extreme outliers for each subject – that is, responses whose RTs were more than 3.5 standard deviations from the given subject's mean– were also excluded (0.32% of correct responses).

The RT data were analyzed in SAS for Windows Release 9.3 (Cary, NC) using mixed-effects regression modeling. This statistical method allows each individual RT from each subject to be entered into one model, without averaging the RTs in a way that would result in a substantial loss of information. Moreover, it allows both item- and subject-level covariates that may influence the pattern of results to be included in the same model. Variables such as frequency and imageability were entered into the model as continuous factors, rather than dichotomized (e.g., as a two-level factor of ‘high’ vs. ‘low’ frequency, as in many previous studies), thereby avoiding loss of power and other problems [73], [74]. Mixed-effects regression models account for subject variability by including the baseline performance (model intercept) of each subject as a random effect. For more complete discussions of this statistical method, see References [81], [82]; for similar analyses, see Reference [68].

In our model, natural logarithm-transformed RT was the dependent variable; imageability, past-tense frequency (natural-log transformed; see above), verb-type (regular vs. irregular) and age-group (child vs. adult) were included as fixed effects. Interactions were specified between age-group, verb-type, and each of frequency and imageability separately, generating separate frequency and imageability coefficients for children and adults, separately for regular and irregular verbs. As in previous work, we included a random effect of subject on the intercept [20]. Significance of all effects was assessed using α = 0.05. All *p*-values are reported as two-tailed. Degrees of freedom were computed using the Satterthwaite approximation.

Fourteen potentially confounding subject- and item-level variables were included as covariates in all analyses. Explicitly including these covariates in the model allows one to directly account for variability attributable to them, which enhances prediction accuracy and decreases the size of the residual error [74]. The fourteen covariates, which are described in detail in Table 1, included two subject-level variables (education and sex), and twelve item-level variables controlling for a range of phonological, semantic and other properties of the verbs (e.g., phonological neighborhood).

**Table 1:** Covariates included in the mixed-effects model.

Covariate	Description
**a) Subject-level**	
*Education*	Years of formal education [101]
*Sex*	Male or female
**b) Item-level**	
Phonological	
*Stem phonological length*	Number of phonemes (with diphthongs counted as one phoneme) in the stem. Phonological length affects working memory; the stem is likely to be held in working memory before production of the past-tense form [20], [77], [102], [103].
*Past-tense phonological length*	Number of phonemes (with diphthongs counted as one phoneme) in the past tense form; longer spoken forms may require more time for syllabification and articulatory planning than shorter ones [20], [104].
*Initial fricative*	A binary variable describing whether the initial sound of the subject's response was a fricative [20], [105].
*Initial plosive*	A binary variable describing whether the initial sound of the subject's response was a plosive [20], [105].
*Phonological neighborhood*	A measure of the frequency of phonologically similar and dissimilar verbs. Calculated from the sum of FK and AP frequency counts (see main text) over all “friends” (i.e., verbs whose past-tense forms rhymed with the past-tense form of the given verb e.g., *sleep-slept* is a friend of *keep-kept)*, minus the sum of the frequencies over all “enemies” (i.e., verbs which do not show this past-tense rhyme similarity, e.g., *spring-sprang* and *bring-brought* are enemies of *fling-flung*). If this difference (which we will refer here to as D) was positive, neighborhood strength was defined as ln(|D|+1), i.e., as the natural log of the absolute value of D; if negative, it was defined as -ln(|D|+1), allowing a verb's neighborhood strength to be negative if it has a preponderance of irregular enemies [77].
*Voicing*	A binary variable describing whether or not the phonemes in the rime of the past-tense form exhibit consistent voicing (e.g., the rime of the regular past-tense *felled* is consistently voiced, as both/l/and/d/are voiced, whereas the rime of the irregular past-tense *felt* is not, as/t/is voiceless). Two voiced phonemes within a coda may be less perceptually distinct, potentially accounting for differences in performance between regular (always consistently voiced) and irregular (not always consistently voiced) verbs [106].
*Phonological changes*	Number of phonological changes between the stem and past-tense form [77].
Semantic and Word-Class	
*Synonym sets*	An estimate of the number of meanings of a given verb [107] computed as the natural logarithm-transformed number of synonym sets (groupings of words that represent one underlying lexical concept) in which the verb appears, based on the synonym sets in WordNet, an on-line database of English [108], [109]
*Noun-to-verb ratio*	An estimate of the likelihood that a given verb has been converted from a noun or into a noun, computed as the natural logarithm of the ratio of each stem form's frequency as a noun to that form's frequency as a verb, based on the combined (FK and AP) frequency counts (see main text) [107]
Other	
*Verb order*	A measure of how many verbs were presented prior to a given verb. Order is likely to be most influential for the first few items, with order effects diminishing rapidly as the subjects become more comfortable with the task; therefore the natural logarithm of item order was used [20], [77].
*Inflectional class of previous verb*	A binary variable describing whether or not the previously presented verb was or was not of the same inflectional class (verb type), i.e., regular or irregular [20].
*Real/novel*	A binary variable describing whether the previously presented verb was real or novel [20], [77].

All fourteen covariates were entered as fixed main effects into the mixed-effects model described above. The covariates were also tested for additional inclusion as random effects in the model [20]. To evaluate whether an item-level covariate should be (additionally) included as a random effect (by subject), which would allow the model to account for differences in the effect of the covariate between subjects, each covariate was separately entered as a random effect into a model that was otherwise identical to the model with the covariates included only as fixed effects. The subject-level covariates were tested in the same way. Any covariate whose inclusion as a random effect resulted in a substantial Akaike's Information Criterion reduction (AIC, a smaller-is-better measure of model fit), as compared to the model with covariates entered only as fixed effects, was retained as a random effect (as well as a fixed effect) in the final mixed-effects model; otherwise it was included only as a fixed effect. Of the fourteen covariates, only verb order improved model fit as a random factor (from AIC = 2118.7 to AIC = 2002.1), and was therefore (additionally) included as such.

## Results

### Children's regulars versus irregulars

Over all children (*n* = 35), examination of the effect of imageability on past tense production response times revealed significant negative coefficients (i.e., the magnitude of the coefficient was significantly greater than zero) both for irregular and for regular past tense forms, with no reliable difference between the coefficients for the two verb types (Figure 1A). That is, significant imageability effects were found for both irregular and regular past-tense forms. Examination of the effect of frequency on response time revealed a significant negative coefficient for irregular past tense forms (i.e., frequency effects were found on irregulars), whereas frequency effects were not observed for regular past tense forms; the difference between the coefficients for the two verb types was significant (Figure 1B).

**Figure 1:** Children's imageability and frequency effects for regular and irregular past-tense forms. In each scatterplot, the line represents the prediction of the mixed effects regression model with regard to the effect of imageability or frequency on the natural logarithm of response times, with the effect of all covariates removed. Points on the graph represent residuals from the model (with the effects of the covariates removed) for the 29 regular and 29 irregular verbs. *B* represents the unstandardized regression coefficient, indicating the slope of the regression line, *t* represents the *t*-statistic of the comparison between *B* and zero, and *p* represents the statistical significance of this comparison.

Thus, the children exhibited imageability effects on irregulars as well as regulars. In contrast, they exhibited frequency effects on irregulars only. The children's lack of frequency effects on regulars does not appear to be explained by confounding statistical or experimental factors. First, it is not explained by ceiling effects on regulars: the RT variance did not differ (as measured by Folded F-tests) between the verb types (*F*(28,28)  = 1.23, *p* = .592). Note also that the mean RTs for regulars and irregulars did not differ (regulars: *M* = 7.80, *SE* = 0.02; irregulars: *M* = 7.79, *SE* = 0.02; *t_1_*(34)  = 0.20, *p* = .841, *t_2_*(56) = 0.21, *p* = .838). Second, it is also not accounted by low power due to smaller sample sizes for regulars. In fact, there were *more* correctly-produced past-tense forms (on which the RT analyses were carried out) for regulars than irregulars (accuracy on regulars: *M* = 97.92%, *SE* = 0.52%; irregulars: *M* = 78.74%, *SE* = 3.66%; *t_1_*(34)  = 10.86, *p*<.0001, *t_2_*(56)  = 5.19, *p*<.0001). Third, as noted above, the regular and irregular verbs were matched on imageability, as well as stem and past-tense frequency. Moreover, fourteen potentially explanatory variables were included as covariates in the regression model, statistically equating regulars and irregulars with regard to various properties.

### Regulars versus irregulars in boys versus girls: Could the inclusion of female subjects explain imageability effects on regulars?

The previous study examining adults' frequency and imageability effects on past tense production revealed sex differences for regulars [20]. In particular, storage (i.e., frequency) effects on regulars were largely due to such effects for women but not men [20]. We therefore examined the possibility that similar sex differences may exist in children; in other words, that the storage (i.e., imageability) effects on regulars observed in the present study may be due to the data from the girls. We thus examined imageability effects on regulars and irregulars in girls versus boys. Likewise, even though no overall frequency effect was found for regulars, we also investigated whether boys and girls differed in frequency effects, as was previously found for adults. To generate separate imageability and frequency coefficients for boys and girls, we added an interaction with sex (male vs. female) to the verb-type by age group by imageability interaction and to the verb-type by age group by frequency interaction in the same model as described above.

#### Imageability effects in girls versus boys

The sex by verb-type by imageability interaction was significant (Figure 2; center box). Girls showed significant imageability effects on regulars, but not irregulars, with the verb-type difference not significant (Figure 2A). In contrast, boys showed significant imageability effects on irregulars, but not regulars, with a significant verb-type difference (Figure 2B). Additionally, the coefficients for irregulars did not differ between the boys and girls, whereas the coefficients for regulars did differ significantly between the sexes (Figure 2; middle row).

**Figure 2:** Children's imageability effects for regular and irregular past-tense forms, by sex. In each scatterplot, the line represents the prediction of the mixed effects regression model with regard to the effect of imageability on the natural logarithm of response times, with the effect of all covariates removed. Points on the graph represent residuals from the model (with the effects of the covariates removed) for the 29 regular and 29 irregular verbs. *B* represents the unstandardized regression coefficient, indicating the slope of the regression line, *t* represents the *t*-statistic of the comparison between *B* and zero, and *p* represents the statistical significance of this comparison.

The observed lack of imageability effects on regulars in boys does not seem to be attributable to confounding factors such as ceiling effects or low power. First, the RT variance in boys did not differ (as measured by Folded F-tests) between regulars and irregulars: *F*(28,28)  = 1.25, *p* = .557. Moreover, boys' mean RTs for regulars and irregulars did not differ (regulars: *M* = 7.757, *SE* = 0.027; irregulars: *M* = 7.786, *SE* = 0.024; *t_1_*(18) = 0.24, *p* = .811, *t_2_*(56)  = 0.80, *p* = .425). Second, boys produced *more* correct past-tense forms for regulars than irregulars (accuracy on regulars: *M* = 97.50%, *SE* = 0.7%; irregulars: *M* = 76.22%, *SE* = 0.38%; *t_1_*(18) = 9.65, *p*<.0001, *t_2_*(56)  = 5.58, *p* = .0001). Finally, note that the same subject- and item-level covariates described above were included in the model used in this analysis.

#### Frequency effects in girls versus boys

The three-way interaction between sex, verb-type and frequency was not significant (Figure 3; center box). For the girls, there was a significant frequency effect for irregulars but not regulars, though the difference between the two verb types was not significant (Figure 3A). For the boys, a negative frequency coefficient for irregulars approached significance, and differed significantly from the coefficient for regulars (which was *positive*, Figure 3B). The coefficients for irregulars did *not* differ between the boys and girls, whereas the coefficients for regulars *did differ* significantly between the sexes (Figure 3; middle row). Over both verb types, frequency effects were found in girls (*B* = −0.017, *t*(5290)  = 2.89, *p* = .004), but not in boys (*B* = −0.001, *t*(5299)  = 0.11, *p* = .915), with a significant difference between them (*B* = −0.017, *t*(5195)  = 2.36, *p* = .018).

**Figure 3:** Children's frequency effects for regular and irregular past-tense forms, by sex. In each scatterplot, the line represents the prediction of the mixed effects regression model with regard to the effect of frequency on the natural logarithm of response times, with the effect of all covariates removed. Points on the graph represent residuals from the model (with the effects of the covariates removed) for the 29 regular and 29 irregular verbs. *B* represents the unstandardized regression coefficient, indicating the slope of the regression line, *t* represents the *t*-statistic of the comparison between *B* and zero, and *p* represents the statistical significance of this comparison.

In summary, examination of potential sex differences among the children indicated that girls but not boys showed imageability effects on regulars, which may largely explain the imageability effects on regulars in the full group of children. Conversely, boys but not girls showed imageability effects on irregulars. We also examined potential sex differences in frequency effects; here, neither girls nor boys showed frequency effects for regulars (although the coefficients for girls and boys were significantly different), while both sexes showed frequency effects for irregulars (these only approached significance for boys, but did not differ from the frequency effects found in girls).

### Further analyses: Comparisons between children and adults

In order to probe for potential developmental changes, we directly compared children's patterns of imageability and frequency effects on regulars and irregulars to the data from adults previously obtained in Prado and Ullman (2009) [20]. Because sex differences were observed here for children (the sex by verb-type by imageability interaction was significant, as were the sex differences in both the imageability and frequency coefficients for regulars), below we examined males and females separately in the comparisons with adults, both for imageability and for frequency effect analyses. (Note that the pattern for adults obtained here was similar to that reported in Prado and Ullman (2009) [20], though the coefficients and *p*-values are slightly different, since the model here included additional data (the children's data) and additional covariates).

#### Imageability effects in children versus adults

For females, the age-group (children vs. adults) by verb-type (regular vs. irregular) by imageability interaction was significant (*B* = −0.070, *t*(5337)  = 2.04, *p* = .041), indicating that the pattern of imageability effects differed between girls and women. Girls showed significantly stronger imageability effects than women on regulars (*B* = 0.070, *t*(5437)  = 3.34, *p*<.001), while on irregulars girls and women did not differ (*B* = 0.001, *t*(5407) = 0.03, *p* = .972). In contrast to girls, women did not show imageability effects for regulars (*B* = 0.006, *t*(5403)  = 0.46, *p* = .648) or for irregulars (*B* = −0.015, *t*(5385)  = 1.08, *p* = .280), and there was no significant difference between the verb types for women (*B* = −0.020, *t*(5334)  = 1.13, *p* = .260).

For males, the age-group by verb-type by imageability interaction was not significant (*B* = 0.004, *t*(5339)  = 0.11, *p* = .915) and the boys and men did not differ in the magnitude of the imageability effect (across both verb types: *B* = 0.021, *t*(5442)  = 1.21, *p* = .225). This indicates that the pattern of imageability effects did not differ between boys and men.

#### Frequency effects in children versus adults

In females, the age-group by verb-type by frequency interaction was not significant (*B* = 0.011, *t*(5430)  = ,0.95 *p* = .344). The age group difference over both verb types (regulars and irregulars) was not significant (*B* = 0.003, *t*(5153)  = 0.38, *p* = .701), indicating that the pattern of frequency effects over both verb types did not differ between girls and women.

In males, the age-group by verb-type by frequency interaction was not significant (*B* = 0.011, *t*(5425)  = 0.93, *p* = .353). The age group difference over both verb types was not significant (*B* = −0.010, *t*(5139)  = 1.57, *p* = .115), indicating that the pattern of frequency effects did not differ between boys and men.

## Discussion

This study examined frequency and imageability effects in the production of (correct) existing English regular and irregular past tense forms in monolingual 8–12 year old children. It additionally directly compared these findings with adult data. The results can be summarized as follows.

Children exhibited imageability as well as frequency effects on irregulars. In contrast, they showed only imageability effects on regulars. When we examined whether the pattern of effects differed between boys and girls, the interaction with sex indicated that the pattern differed by sex for imageability effects but not frequency effects (central panels of Figures 2 and 3). Specifically, boys and girls differed significantly in imageability effects on regulars, with only girls showing such effects. In contrast, boys and girls did not differ significantly in imageability effects on irregulars (Figure 2). For frequency effects, the sex by verb-type interaction was not significant, though over both verb types, girls but not boys showed frequency effects.

Within-sex comparisons between children and adults indicated that with regard to imageability effects, females but not males showed age-group differences. Specifically, for females, imageability effects were found only on regulars and only in girls – that is, not on irregulars in either age group, and not in women in either verb type. For frequency, no age group differences were observed in either males or females.

The following pattern emerges from the data (see Table 2). For females, between childhood and adulthood imageability effects on regulars disappear. In contrast, frequency effects on regulars in females do not change reliably during this period (the frequency coefficients were not significantly different between girls and women), though the frequency effect reaches significance (it is reliable) in women [20], but not in girls (Figure 3). For irregulars, the pattern does not change from childhood to adulthood: both girls and women show frequency effects and neither shows imageability effects.

**Table 2:** Summary of frequency and imageability effects, by verb type, sex and age group.

	Regular Past Tenses		Irregular Past Tenses	
	Frequency Effects	Imageability Effects	Frequency Effects	Imageability Effects
Boys	NO	NO	YES*	YES
Men	NO	NO	YES	YES
Girls	NO	YES	YES	NO
Women	YES	NO	YES	NO

*Approaching significance.

Note: The results for men and women are from Prado & Ullman (2009:861) [20].

Males exhibited a somewhat different pattern. For regulars, neither frequency nor imageability effects change from childhood to adulthood; no effects of either type were found in either age group (Table 2). Likewise, for irregulars, the pattern of effects does not change reliably with age. Here, however, both boys and men show imageability effects; frequency effects also do not differ significantly between boys and men, though they reach significance only in men (approaching significance in boys).

This pattern of results does not appear to be explained by confounding experimental or statistical factors: the findings are not explained by ceiling effects, by differences in power, or by numerous item- and subject-level covariates. Note also that the sex differences in imageability effects on regulars cannot be attributed to potential sex differences in reading levels, since the boys and girls in this study did not differ in reading abilities (see Methods).

Given the different interpretations of the lack of frequency effects (and potentially of imageability effects) under single-mechanism and dual-system frameworks, we discuss the results separately from the two perspectives.

Within a single-mechanism framework, all inflected forms – regular and irregular – are expected to depend on stored representations in all subjects: that is, in children and adults, and in both sexes. Therefore, the significant frequency effects found in the full group of children on irregulars are expected in this view. The significant imageability effects on irregulars in the full group of children could presumably also be accounted for, although it is important to point out that, to our knowledge, imageability has not thus far been considered in connectionist models of inflectional morphology. Children's lack of frequency effects on regulars might be argued to be due to the contribution of neighboring (i.e., phonologically similar) verbs to the memory traces of regular forms overwhelming the contribution of each verb's individual past tense frequency (see Introduction). However, our inclusion of phonological neighborhood as a covariate (see Table 1) suggests that phonological consistency might not explain the lack of frequency effects on regulars. Finally, although the observed pattern of sex differences on imageability effects might potentially be explainable by single-mechanism models, to our knowledge such models have not thus far addressed such differences (for additional discussion, also see [20]). Thus, it remains to be seen whether future connectionist models can accommodate the findings reported here.

Within a dual-system framework, irregular inflected forms are expected to be stored by all language users. Based on prior results, regular inflected forms may tend to be stored by women, but not men [20]. One possibility is that children follow this adult pattern. Indeed, boys do show the same pattern as men, lacking both frequency and imageability effects on regulars, but showing evidence of both imageability and frequency effects on irregulars. This suggests that, just like men, boys compose regulars but store irregulars. Girls show a somewhat different pattern. For irregulars, girls show the same pattern as women, with frequency but not imageability effects; the frequency effects indicate the storage of irregularly inflected forms. However, girls do not show the same pattern as women for regulars: girls show imageability effects but not frequency effects, whereas women show the opposite pattern. This suggests that girls, like women, store regulars, but the lexical properties that influence this storage change over the course of development.

Here we suggest that the overall pattern of results reflects three different principles. First, we suggest a developmental trajectory in which imageability precedes frequency as a mechanism facilitating the storage of inflected forms. This interpretation is supported by several lines of evidence. Previous findings indicate that reliance on imageability (including with regard to language) *decreases* between childhood and adulthood; in other words, children rely more on imageability than adults [48], [83], [84]. At the same time, it is plausible that frequency *increasingly* influences memory traces between childhood and adulthood. That is, frequency may play a larger (i.e., more significant) role in lexical access with increasing exposure to language. In this view, over time, as increasing exposure to words strengthens the memory traces for those forms, frequency plays an increasingly important explanatory role in lexical access. Additionally, it is plausible that over the course of development, the frequency (exposure) distribution of words experienced by a given individual will increasingly (i.e., as the signal outweighs the noise) reflect the more general frequency distribution in the population (which is measured by frequency counts), leading to increasing frequency effects with time. The notion that frequency effects have an increasing influence during development is further supported by previous findings which overall suggest more sporadic frequency effects on past tenses in children as compared to adults, even for irregulars (see Introduction).

Second, girls may tend to develop language skills earlier than boys [85]–[91]. Indeed, brain areas involved in language appear to develop earlier in girls than boys [90], [91]. More generally, females (girls as well as women) have been argued to have superior verbal skills than males [21]–[25], [92]. Since the influence of frequency may be more intrinsically dependent on language skills than imageability (e.g., the former crucially depend on linguistic forms, whereas the latter rely heavily on semantics), the storage of linguistic forms may be influenced earlier and more strongly by frequency (but perhaps not by imageability) in females than males. Conversely, since males (both boys and men) may tend to have advantages over females at visuo-spatial processing [23], [93], [94] imageability (but not frequency) may play an earlier and perhaps larger explanatory lexical access role in males than females.

Third, the storage of irregular inflected forms may depend more on frequency than regular inflected forms. Since irregulars can only be stored, every encounter with an irregular past-tense form should influence its storage; frequency would thus play an important role for irregulars earlier on than for regulars (which may be either stored or composed).

Together, these three principles may explain the pattern of results observed here. For irregular past tenses, girls may already show a significant effect of frequency, which may thus explain a substantial degree of the variability in the access of these forms, leaving imageability (and perhaps other factors) with little explanatory power – especially if the influence of imageability is not particularly strong in girls due to the status of their visual-spatial skills. In other words, 8-12 year old girls may have already shifted from imageability to frequency as a factor facilitating the storage of these forms. For regular past tenses, girls also tend to rely on storage (e.g., due to their memory advantages; see below), but still depend on imageability as a means to do so, in line with the expectation that regulars undergo the shift to frequency later than irregulars. However, by adulthood, women should have transitioned from imageability to frequency as the dominant mechanism underlying access, even for regulars, as we suggest younger girls have already done for irregulars. Thus women show frequency effects but not imageability effects for both verb types.

For males, the story is somewhat different. On irregulars, boys show reliable imageability effects, whereas their frequency effects do not reach significance. This is consistent with strong visuo-spatial skills and weaker verbal skills in boys (as compared to girls), leading to strong imageability effects but the slower development of frequency effects. Note that the imageability and frequency effects may also affect each other: the weaker frequency effects are less likely to overwhelm imageability effects, while strong imageability effects may further weaken the effect of frequency. By adulthood, men still show imageability effects on irregulars, even though they have developed clear frequency effects by this point. Again, this is consistent with strong visuo-spatial skills in males as well as weaker verbal skills, even though the cumulative effect of frequency is strong enough to lead to significant frequency effects. For regulars, there is no indication of any storage for either boys or men. One possibility is that adult men are delayed even relative to young girls in their reliance on memory for these forms. However, this seems implausible, since the men ranged in age from 18 to 50. Alternatively, males and females may tend to have different computational strategies for regular forms, both as children (at least around age 10) and as adults. On this view, females often store regulars, while males tend to rely on composition, with this sex difference likely due in part to a lexical memory advantage for females [20], [25].

Overall, within a dual system framework, the results from the current study provide further support for a model in which irregular inflected forms are always stored, whereas regular inflected forms may be composed, but can also be stored, with various item- and subject-level factors modulating their storage vs. composition [14], [92], [95]. Moreover, the present study has revealed for the first time a developmental trajectory that is at least somewhat different for boys and girls.

## Conclusion

This study was designed to contribute to our understanding of the distinction between the storage and composition of complex linguistic forms. Specifically, it attempted to fill an existing gap concerning frequency and imageability effects on regular and irregular inflected forms in children. The findings suggest that 8–12 year old children store irregulars more reliably than regulars. However, the pattern of storage is also influenced by sex. Boys show evidence of storage for irregulars but not regulars, while girls show evidence of storage for both. Additionally, boys seem to rely particularly on imageability and girls particularly on frequency for lexical storage and access. Although not ruling out single-mechanism models, the new child data are compatible with a dual-system view in which idiosyncratic (unpredictable) forms, such as irregular inflected forms, are stored, whereas rule-governed forms, such as regular inflected forms, can be either composed or stored, with storage a function of various factors. The findings also indicate that there is a developmental shift in the basis of storage between the age range studied (8–12) and adulthood. Imageability may play a greater role in the memorization of inflected words in children than adults, whereas frequency may play a greater role in the memorization of inflected forms in adults than children, a finding which will need to be confirmed in future studies.

The current findings make a number of contributions to the previous literature on frequency effects on inflected forms in children. First, this study demonstrates the utility of mixed effects modeling in this area of investigation. Because of the improved methodology used here, the present results strengthen previous reports of frequency effects on children's processing of irregular but not regular forms [58], [65]. As the first study to examine imageability in addition to frequency effects in children's processing of inflected forms, this study builds on previous work by providing further insight into the bases of lexical storage in children. The findings additionally corroborate recent acquisition evidence regarding a link between imageability and inflected forms; this evidence indicates that children acquire inflected (plural) forms earlier in development for higher imageability than lower imageability nouns [96]. Taken together, these different lines of research provide growing evidence regarding the relation between imageability and inflected forms from both acquisition and processing. Most importantly, the current study contributes several new discoveries to the field of child language, including the findings that regulars can to some extent be stored in children (as well as adults), that there appear to be sex differences with regard to storage effects in children (as well as adults), and that the bases of storage of inflected forms appears to change to some degree between childhood and adulthood.

The present investigation has also brought to light some novel predictions and directions for future research. For example, imageability effects on irregulars were reliable in males but not in females. Because irregulars (unlike regulars) *must* rely on stored representations in all theoretical frameworks [50], this pattern may be taken as evidence that imageability has a stronger influence on lexical storage in males than females, perhaps due both to strong visuo-spatial skills in males and strong verbal skills in females. Note that a stronger influence of imageability in males than females leads to an interesting prediction, namely that the often observed pattern of imageable (concrete) words being acquired earlier by children than abstract (less imageable) words [37], [80], [97]–[100] may hold more strongly for boys than for girls. In contrast, girls may perhaps learn abstract words earlier than boys. To our knowledge, these predictions have not yet been examined.

Finally, it is important to keep in mind that this study examined only 8–12 year old children and adults. Nevertheless, it is not unreasonable to extrapolate from the patterns of frequency and imageability effects in the two age groups. In particular, intermediate age groups (e.g., adolescents) should show similar frequency and imageability patterns as the two age groups where they did not differ, or intermediate patterns where they did. However, it is difficult to extrapolate to younger (e.g., toddlers) or older (e.g., the elderly) age groups. Thus the influence of frequency, imageability and sex in younger and older age groups warrants examination in future studies. Likewise, the present investigation focused solely on inflectional morphology, in particular on English past tense. Future studies should investigate whether the current results might generalize to other tasks (e.g., [6]), other inflectional paradigms, other languages, and other aspects of language, including derivational morphology and syntax.
